# Thiolated chitosan-modified PLA-PCL-TPGS nanoparticles for oral chemotherapy of lung cancer

**DOI:** 10.1186/1556-276X-8-66

**Published:** 2013-02-09

**Authors:** Liqin Jiang, Xuemin Li, Lingrong Liu, Qiqing Zhang

**Affiliations:** 1 Tianjin Key Laboratory of Biomaterial Research, Institute of Biomedical Engineering, Peking Union Medical College & Chinese Academy of Medical Sciences, Tianjin, 300192, China

**Keywords:** Oral chemotherapy, PLA-PCL-TPGS, Thiolated chitosan, Nanoparticles, Lung cancer

## Abstract

Oral chemotherapy is a key step towards ‘chemotherapy at home’, a dream of cancer patients, which will radically change the clinical practice of chemotherapy and greatly improve the quality of life of the patients. In this research, three types of nanoparticle formulation from commercial PCL and self-synthesized *d*-α-tocopheryl polyethylene glycol 1000 succinate (PLA-PCL-TPGS) random copolymer were prepared in this research for oral delivery of antitumor agents, including thiolated chitosan-modified PCL nanoparticles, unmodified PLA-PCL-TPGS nanoparticles, and thiolated chitosan-modified PLA-PCL-TPGS nanoparticles. Firstly, the PLA-PCL-TPGS random copolymer was synthesized and characterized. Thiolated chitosan greatly increases its mucoadhesiveness and permeation properties, thus increasing the chances of nanoparticle uptake by the gastrointestinal mucosa and improving drug absorption. The PLA-PCL-TPGS nanoparticles were found by FESEM that they are of spherical shape and around 200 nm in diameter. The surface charge of PLA-PCL-TPGS nanoparticles was reversed from anionic to cationic after thiolated chitosan modification. The thiolated chitosan-modified PLA-PCL-TPGS nanoparticles have significantly higher level of the cell uptake than that of thiolated chitosan-modified PLGA nanoparticles and unmodified PLA-PCL-TPGS nanoparticles. *In vitro* cell viability studies showed advantages of the thiolated chitosan-modified PLA-PCL-TPGS nanoparticles over Taxol® in terms of cytotoxicity against A549 cells. It seems that the mucoadhesive nanoparticles can increase paclitaxel transport by opening tight junctions and bypassing the efflux pump of P-glycoprotein. In conclusion, PLA-PCL-TPGS nanoparticles modified by thiolated chitosan could enhance the cellular uptake and cytotoxicity, which revealed a potential application for oral chemotherapy of lung cancer.

## Background

Lung cancer continues to be one of the most common fatal cancers worldwide. Oral chemotherapy is quickly emerging as an appealing option for cancer patients because it is less stressful, being that the patient will have less hospital visits and can still maintain a close relationship with health care professionals [1]. These features make oral delivery especially attractive for mass immunization and self-administration of medications. In addition, oral chemotherapy could maintain a sustained moderate concentration of the drug in the circulation to achieve a prolonged exposure of cancerous cells to the drug as well as to avoid high peak above maximum tolerable concentration. This will increase the therapeutic efficacy and decrease the side effects. However, most anticancer drugs especially those with excellent antitumor effects such as paclitaxel are poorly bioavailable. This is because oral administration of taxoids (paclitaxel and docetaxel) presents an extremely low bioavailability, with a less than 1% extent of oral absorption [2,3]. The low systemic exposure of oral paclitaxel is, at least in part, due to their high affinity for P-glycoprotein (P-gp) multidrug efflux pump in the mucosa of the gastrointestinal (GI) tract [4,5]. P-gp in the mucosa of the gastrointestinal tract may limit the absorption of the orally administered taxanes and mediate their direct excretion into the intestinal lumen [5]. First-pass metabolism by cytochrome P450 isoenzymes in the gut wall and/or in the liver may also play a role in the low oral bioavailability of paclitaxel and docetaxel [6,7]. Alternative pharmaceutical methods to improve oral bioavailability of taxoids and other antitumor agents are currently under intense investigation [2,8-10]. The general medical approach is to make use of P-gp/P450 inhibitors such as cyclosporine A to suppress the elimination process [9,10]. However, cyclosporine A may cause severe damage to the immune system of the body and, thus, create severe complications during cancer treatment. Polymeric nanoparticles are highly attractive from the pharmaceutical point of view due to their desirable properties such as biocompatibility, biodegradability, and controlled release. Furthermore, polymeric nanoparticles could avoid recognition by the P-gp efflux pump and, thus, have a strong potential to enhance the oral bioavailability of poorly absorbed drugs [11-13]. Their small size and their large specific surface area favor their absorption compared to larger drug carriers. In addition, polymeric nanoparticles can protect encapsulated drugs from luminal degradation as well as gut-wall metabolism [8]. Moreover, they could reduce the multi-drug resistance (MDR) that characterizes many anticancer drugs by a mechanism of internalization of the drug, reducing its efflux from cells mediated by the P-gp. It seems to be commonly accepted that particle surface properties are utmostly important for their uptake by intestinal epithelial cells. Therefore, many methodologies and innovative techniques have been developed to enhance the intestinal absorption of particles, either by altering their surface properties or by conjugating a targeting molecule at their surface [14]. In this research, our group proposed a new type of polymeric nanoparticles, i.e., biodegradable poly(lactide-*coε*-caprolactone)-d-α-tocopheryl polyethylene glycol 1000 succinate (PLA-PCL-TPGS) nanoparticles modified with thiolated chitosan for oral chemotherapy using paclitaxel as a therapeutic agent due to its high therapeutic efficacy against a broad spectrum of tumors and its great commercial success as one of the best-selling antitumor therapeutic drugs.

Chitosan, a linear polysaccharide derived from chitin obtained from crustacean shells, has emerged as a useful drug delivery matrix because of it polycationic nature, biodegradability, biocompatibility, mucoadhesiveness, and ease of physical and chemical modification [15]. The interaction between cationic amino groups on chitosan and anionic moieties such as sialic and sulfonic acids on the mucus layer is responsible for its mucoadhesiveness [16]. In addition, chitosan enhances epithelial permeability through the opening of tight junctions between epithelial cells [17]. Recently, it was reported that the covalent attachment of thiol groups to polymers greatly increases their mucoadhesiveness and permeation properties without affecting biodegradability [16,18]. Thiolated chitosan-modified nanoparticles are expected to be appropriate carriers for oral absorption of drugs [19-21]. Thiolated chitosan has many advantages as a carrier in nanoparticulate drug delivery systems. It is nontoxic, biocompatible, and biodegradable and has been proven to control the release of drugs, proteins, and peptides. It is soluble in aqueous media, avoids the use of organic solvents, and does not require further purification of nanoparticles [22]. Thus, thiolated chitosan was used in the present study to be absorbed on the nanoparticle surface by electrostatic forces of attraction between positive and negative charges. In this research, PLA-PCL was used to maintain the desirable mechanical strength of the polymer. Vitamin E *d*-α-tocopheryl polyethylene glycol 1000 succinate (Vitamin E TPGS, or simply TPGS) is a water-soluble derivative of naturally sourced vitamin E, which is formed by esterification of vitamin E succinate with polyethylene glycol 1000. Previous studies revealed that TPGS was able to improve drug permeability across biological membranes by inhibition of P-gp pumps and, thus, increase the drug absorption capability and decrease P-gp-mediated MDR in cancer cells [23-25]. In addition, TPGS was able to effectively inhibit the growth of human lung cancer cells in cell culture and in animal models [26]. The superior antitumor activity of TPGS is mainly due to its increasing ability to induce apoptosis in tumor cells [26-28]. A few studies have shown synergistic effects of combinations of TPGS with other antitumor drugs [27]. Furthermore, it has been found that TPGS-emulsified nanoparticles had higher encapsulation efficacy and cellular uptake, longer half-life, and higher therapeutic efficiency of the formulated drug than those emulsified by poly(vinyl alcohol), a commonly used emulsifier in nanoparticle formulation process [24]. Thus, we were inspired to fabricate a novel thiolated chitosan-modified PLA-PCL-TPGS nanoparticle as oral anticancer drug carrier for lung cancer chemotherapy. The chemical structure of PLA-PCL-TPGS random copolymer is shown in Figure 1[24].

**Figure 1:** **Chemical structure and ^1^H-NMR spectra of PLA-PCL-TPGS copolymer. **(**A**) Chemical structure of PLA-PCL-TPGS copolymer; (**B**) typical ^1^H-NMR spectra of PLA-PCL-TPGS copolymer.

## Methods

### Materials

d,l-lactide (3,6-dimethyl-1,4-dioxane-2,5-dione, C_6_H_8_O_4_) and *d*-α-tocopheryl polyethylene glycol 1000 succinate (C_33_O_5_H_54_ (CH_2_CH_2_O)_23_) were purchased from Sigma-Aldrich (St. Louis, MO, USA). *ε*-caprolactone (CL) were obtained from Acros Organics (Geel, Belgium). Thiolated chitosan (Mw 33000 Da) was from NanoMed Biotech Co. Ltd (Shenzhen, China). Poly(ε-caprolactone) (PCL) (MW 42000 Da), and stannous octoate (Sn(OOCC_7_H_15_)_2_) were also purchased from Sigma (St. Louis, MO, USA). Paclitaxel powder of purity 99.9% was from BioOne Biotech Co. Ltd (Shenzhen, China). Fetal bovine serum was received from Gibco (Life Technologies, AG, Switzerland). Methanol and acetonitrile were obtained from EM Science (Mallinckrodt Baker, USA). Deionized (DI) water produced by Millipore Water Systems (Millipore Corporation, Billerica, USA) was utilized throughout all experiments.

### Synthesis and characterization of PLA-PCL-TPGS random copolymer

PLA-PCL-TPGS random copolymers were synthesized from *ε*-caprolactone, lactide, and TPGS in the presence of stannous octoate as a catalyst via ring opening polymerization. In short, pre-weighted amounts of *ε*-caprolactone, lactide, TPGS, and one drop of stannous octoate were added in a flask. The mixture was heated to 145°C and allowed to react for approximately 16 h. Synthesis was carried out under an oxygen- and moisture-free environment. The product was dissolved in dichloromethane (DCM) and then precipitated in excess cold methanol to remove unreacted monomers and TPGS. The final product was collected by filtration and dried under vacuum. The TPGS content and number-averaged molecular weight of the copolymer was determined by ^1^H NMR in CDCl_3_ at 300 Hz (Bruker ACF300, Bruker AXS Pte Ltd., Singapore).

### Preparation of thiolated chitosan-modified paclitaxel-loaded nanoparticles

Nanoparticles were prepared by a modified solvent extraction/evaporation technique [29,30]. In brief, 11 mg of paclitaxel powder and 100 mg of PLA-PCL-TPGS copolymer were weighed and dissolved in 6 ml DCM. The organic solution was immediately poured into 100 ml of 0.03% (*w*/*v*) TPGS solution under mild stirring. The mixture was then sonicated for 90 s at 30 W output to form water-in-oil emulsion. The emulsion was further evaporated under ambient conditions overnight to remove DCM. The nanoparticles were harvested by centrifugation at 80,000×*g* for 15 min and then washed three times to remove the emulsifiers and unentrapped drug. The resulting nanoparticles were finally resuspended in 5 ml of deionized water and lyophilized. The PLA-PCL-TPGS nanoparticles was further modified by thiolated chitosan using a method described previously [31]. Preweighed thiolated chitosan was dissolved in deionized water at a concentration of 0.5 mg/ml. The nanoparticles were suspended in thiolated chitosan solution at a concentration of 9.5 mg/ml by sonication at 30 W power output for 30 s in an ice bath, and then were collected by centrifugation at 80,000×*g* for 15 min. The coumarin-6-loaded nanoparticles were prepared by encapsulation of 0.1% (*w*/*v*) coumarin-6 instead of paclitaxel. Thiolated chitosan-modified PCL nanoparticles were fabricated by the same procedure.

### Characterization of nanoparticles

#### Particle size and zeta potential

Particle size and size distribution of nanoparticles were measured using dynamic light scattering on a Malvern Zetasizer Nano-ZS90 (Malvern Instruments, Worcestershire, UK). The lyophilized nanoparticles were diluted with DI water before measurement. Surface charge of the nanoparticles was determined by laser Doppler anemometry using a Zetasizer Nano Series (Malvern Instruments). All measurements were done in triplicate.

#### Surface morphology

The morphology of nanoparticles was characterized by field emission scanning electron microscopy (FESEM; ZEISS 77 SUPRA 40VP, Carl Zeiss, Co., Ltd., Shanghai, China) at 5.0 kV electron high tension. To prepare samples for the FESEM observations, a drop of the particle suspension was placed on a grid or a stud, and the supernatant liquid was removed with a capillary after the particles were allowed to settle. The particles were then coated with platinum layer for 30 s.

#### Drug loading and encapsulation efficiency

The encapsulation efficiency (EE) and the actual drug loading of the nanoparticles were measured by high-performance liquid chromatography (LC 1100, Agilent Technologies, Santa Clara, USA) as described before [31,32]. In short, dried nanoparticles (5 mg) were dissolved in 1 ml of methylene chloride under vigorous vortex. The organic solution was transferred to 5 ml of mobile phase consisting of acetonitrile and deionized water (50:50, *v*/*v*). Methylene chloride was evaporated under a nitrogen stream until a clear solution obtained. The samples were then used for high-performance liquid chromatography (HPLC) analysis. The column effluent was monitored at 227 nm with a UV–vis detector. The standard size HPLC column (4.6 × 250 mm) is run at a flow rate of 1 mL/min. The drug encapsulation efficiency was defined as the percentage of the drug loaded in the final product. All these experiments were done in triplicates.

#### In vitro drug release

Accurately weighted aliquots of drug-loaded nanoparticles (15 mg) were suspended in 5 ml release medium (PBS pH 7.4 containing 0.1% *w*/*v* Tween 80). The use of Tween 80 in the release media was able to increase the solubility of drug in the PBS and avoided the binding of drug to the tube wall. The nanoparticle suspension was transferred into a dialysis tubing membrane which is sealed at one end with a clamp. The sealed dialysis bag was placed into a centrifuge tube and immersed in 15-ml release medium. The centrifuge tube was placed in an orbital water bath shaking at 130 rpm at 37.0°C. A 10 ml aliquots of samples was periodically removed for HPLC analysis and replaced with fresh medium. The samples were extracted with 2 ml methylene chloride and reconstituted in 5 ml mobile phase. Methylene chloride was evaporated under a nitrogen stream until a clear solution was obtained. The analysis procedure was the same as for the determination of drug EE.

#### In vitro cellular uptake of nanoparticles

Caco-2 cells which were obtained from the American Type Culture Collection (Manassas, USA) were used in this research to simulate the gastrointestinal barrier for oral chemotherapy. The cells were grown in tissue culture flasks maintained at 37°C in a humidified, 5% CO_2_ atmosphere. The medium, Dubelco's modified essential medium (DMEM) supplemented with 100 μg/ml streptomycin and 20% fetal bovine serum, was freshened once every 3 days. After reaching 70% to 90% confluence, the cells were harvested with 0.25% of trypsin-EDTA solution (Invitrogen, Corporation, Grand Island, USA) and cultured in 96-well black plate (Corning Inc., Corning, USA) at the density of 1.3 × 10^4^ cells per well; when the cells reached confluence, the cells were equilibrated with HBSS buffer at 37°C for 60 min and then incubated with coumarin-6-loaded nanoparticle suspension medium. The nanoparticles were well-dispersed in the culture medium at concentrations of 100, 250, and 500 μg/ml. Nanoparticle dispersions were incubated at 37°C in a 5% CO_2_ atmosphere for 2 h. After incubation with the corresponding nanoparticles, the suspension was removed from the wells, and the cell monolayers were rinsed three times with 50 μl cold PBS (pH 7.4) to remove any traces of nanoparticles left in the wells. After that, the cells were lysed with 50 μl of 0.5% (*w*/*v*) Triton-X 100 in 0.2 N NaOH solution (Sigma-Aldrich, MO, USA). The fluorescence intensity presented in each well was then measured on a GENios Lueifcrase microplate reader (Tecan Group Ltd., Männedorf, Switzerland) with excitation wavelength at 430 nm and emission wavelength at 485 nm. Cellular uptake efficiency was expressed as the percentage of cell-associated fluorescence vs. that present in the positive control. Culture of human lung cancer cell lines A549 cells and their uptake of the coumarin-6-loaded nanoparticles were performed using the same procedure.

Caco-2 cells were reseeded in the Lab-Tek chambered cover glass system (Nalge Nunc International, Rochester, USA). After the cells were incubated with 250 μg/ml coumarin-6-loaded thiolated chitosan-modified PLA-PCL-TPGS particle suspension at 37°C for 2 h, the cells were rinsed with cold PBS buffer for three times and then fixed with 70% ethanol solution for 20 min. The cells were further rinsed twice with PBS and then counter-stained with 4′,6-diamidino-2-phenylindole dihydrochloride (DAPI; Fluka, Buche, Switzerland) for the visualization of the cell nuclei. The cell monolayer was rinsed twice with PBS solution and mounted using the Dako fluorescent mounting medium (Dako, Carpinteria, USA) to be observed by confocal laser scanning microscope (CLSM; Olympus Fluoview FV-1000, Olympus Optical. Co., Ltd., Tokyo, Japan). The images of the cells were determined with differential interference contrast channel, and the images of coumarin-6-loaded nanoparticles and the nuclei of the cells stained by DAPI were recorded with the following channels: blue channel (DAPI) with excitation at 340 nm and green channel (coumarin-6) with excitation at 488 nm.

#### Cell viability assay

A549 cells were counted and seeded in 96-well plates at a density of 0.5 × 10^4^ cells per well and incubated overnight to allow cell attachment. The cells were incubated with drug-loaded PLA-PCL-TPGS nanoparticle suspension, thiolated chitosan-modified PLA-PCL-TPGS nanoparticles, and Taxol® (Bristol-Myers Squibb, New York, USA) at 0.25, 2.5, 12.5, and 25 μg/ml equivalent paclitaxel concentrations and blank thiolated chitosan-modified PLA-PCL-TPGS nanoparticles with the same amount of nanoparticles for 24, 48, and 72 h, respectively. At the determined time, the formulations were replaced with fresh DMEM containing MTT (5 mg/ml), and the cells were then incubated for additional 4 h. MTT-containing medium was aspirated off, and 150 ml of DMSO was added to dissolve the formazan crystal formed by living cells. The absorbance at 570 nm was measured by a microplate reader (Model 680, Bio-Rad Laboratories, Hertfordshire, UK). Untreated cells were taken as a control with 100% viability, and cells without the addition of MTT were used as blank to calibrate the spectrophotometer to zero absorbance. IC50 values (concentration required to reduce cells viability by 50% as compared to the control cells) for each sample was calculated by curve fitting of the cell viability data. The results are expressed as mean ± SD of one representative experiment performed in triplicate, and the experiments were performed three times.

#### Ex vivo study

The everted sac method was chosen for the measurement of transportation of paclitaxel across the intestine barrier. It was carried out according to the slightly modified method that was described previously [33], as follows.

First, a section of about 5 cm of the jejunum was removed from a male rat under ketamine (50 mg/kg) and chlorpromazine (10 mg/kg) anesthesia and washed with Krebs-Ringer bicarbonate solution of pH = 7.4. This section was then gently inverted with a glass rod, and a tube was inserted in one side of the section and tied securely with tape. The other side of the intestine was tied, and 1 mL Krebs-Ringer bicarbonate solution was poured through the hypodermic needle in the tube. The gut sac was placed in a medium saturated with 95% O_2_, 5% CO_2_, and contained the test sample in Krebs-Ringer bicarbonate solution at 37°C. The test samples used include: (1) paclitaxel (1 mg) as Taxol®, and (2) thiolated chitosan-modified PLA-PCL-TPGS nanoparticles (equivalent to 1 mg of paclitaxel). In absorption studies, an O_2_ and CO_2_ mixture was bubbled into the intestinal mucosa to obtain intestinal peristaltic movement. At certain periods of time, 0.5-mL samples were drawn from inside the intestine and replaced with the same volume of fresh medium. The amount of transported paclitaxel in the samples was measured by the HPLC method.

#### Statistical analyses

Data were presented as the mean ± SD. Student's *t* test was used to assess the differences between means. A *P* value <0.05 was considered to indicate a significant difference.

## Results and discussions

Synthesis and characterization of PLA-PCL-TPGS random copolymer.

The structure of the synthesized PLA-PCL-TPGS copolymer was detected by ^1^H NMR in CDCl_3_. Figure 1 shows the chemical structure of PLA-PCL-TPGS random copolymer and ^1^H NMR spectroscopy of the PLA-PCL-TPGS copolymer. The signals at 5.2 and 1.69 ppm (peaks a and e) were assigned to the CH protons and methyl protons -CH_3_ of PLA segment, respectively. The peak at 3.65 ppm (peak c) was assigned to the -CH_2_ protons of PEO part of TPGS. The lower peaks in the aliphatic region belong to various moieties of vitamin E tails. The peaks at 4.06 (peak b), 2.31 (peak d), 1.60 to 1.70 (peak e), and 1.35 to 1.43 (peak f) were assigned to -OCH_2,_ -COCH_2,_ -CH_2_ (4 H), and -CH_2_ (2 H) segments of PCL, respectively [24]. The molecular weight of the PLA-PCL-TPGS was calculated using the ratio between the peak areas at 4.06 (peak area 9.64), 5.2 (peak area 1.23), and 3.65 (peak area 3.00). The number-averaged molecular weight of the PLA-PCL-TPGS random copolymer was determined to be 33,229. The feeding ratios of *ε*-caprolactone, lactide, and TPGS molecular mass were 75%, 15%, and 10%, respectively. However, the ratios of *ε*-caprolactone, lactide, and TPGS molecular mass which were integrated into the PLA-PCL-TPGS copolymers were 87.18%, 8.17%, and 4.64%.

### Characterization of nanoparticles

#### Size, zeta potential, and encapsulation efficiency

The particle size data of the 5% thiolated chitosan-modified PCL nanoparticles (CNP), unmodified PLA-PCL-TPGS nanoparticles (UNP), 5% thiolated chitosan-modified PLA-PCL-TPGS nanoparticles (TNP), and 20% thiolated chitosan-modified PLA-PCL-TPGS nanoparticles (DNP) fabricated in this research are presented in Table 1. The particle size was found to be an important parameter regarding particle uptake. The small nanoparticle size may provide a large surface area and increase in mucin adsorption, which leads to a high mucoadhesive property for the nanoparticles [34]. The permeability of the particles through the intestinal mucosa decreases with increasing particle size reaching a cut-off at around 500 nm [35,36]. The average diameter of the resulted nanoparticles was around 200 nm, which is in the size range favoring the intestinal uptake of the nanoparticles [2,8]. The results also showed that the addition of thiolated chitosan resulted in a slight increase in particle size. Zeta potential analysis confirmed that surface modification with 5% thiolated chitosan reversed the PLA-PCL-TPGS nanoparticles from a negative surface charge of −18.29 mV to a significantly positive charge of +24.66 mV. As reported in the literature, positive surface charge could enhance the mucosal uptake due to anionic nature of mucous layer [37].

**Table 1:** Effects of thiolated chitosan modification on size, encapsulation efficiency, and zeta potential

**Group**	**Polymer**	**Size (nm)**	**PDI**	**Zeta potential (mV)**	**Drug content (%)**	**EE (%)**	**Thiolated chitosan modification**
CNP	PCL	203.56 ± 4.35	0.335	−19.63 ± 4.10	8.69	86.55	5%
UNP	PLA-PCL-TPGS	198.46 ± 2.49	0.246	−18.29 ± 3.25	9.89	98.79	None
TNP	PLA-PCL-TPGS	206.15 ± 3.66	0.286	24.66 ± 4.19	9.79	97.56	5%
DNP	PLA-PCL-TPGS	219.33 ± 4.25	0.317	26.18 ± 5.02	9.88	98.55	20%

*PDI* polydispersity index; *EE* drug entrapment efficiency; *n* = 3.

Regarding the drug EE, it can be seen from Table 1 that the 5% thiolated chitosan-modified PLA-PCL-TPGS nanoparticles achieved much higher EE than the 5% thiolated chitosan-modified PCL nanoparticles. This might be contributed to the self-emulsification effect of TPGS segment in the PLA-PCL-TPGS copolymer [2,8].

#### Surface morphology

Surface morphology of the 5% thiolated chitosan-modified PLA-PCL-TPGS nanoparticles was inspected by FESEM. Figure 2 shows the FESEM image of 5% thiolated chitosan-modified PLA-PCL-TPGS nanoparticles. The FESEM image further confirmed the particle size determined by laser light scattering. The morphology of the nanoparticles exhibited well-formed spherical shape with rough surface.

**Figure 2:** FESEM image of paclitaxel-loaded 5% thiolated chitosan-modified PLA-PCL-TPGS nanoparticles.

#### In vitro drug release assay

The *in vitro* drug release profiles of the CNP, UNP, and TNP in the first 32 days are presented in Figure 3. The drug release from the TNP was found to be 38.47% and 66.59% of the encapsulated drug in the first 5 days and after 32 days, respectively, which was much faster than the CNP, which was only 20.10% and 38.00%, respectively, in the same periods. The faster drug release of TNP may be attributed to the lower molecular weight and the higher hydrophilicity of PLA-PCL-TPGS copolymer in comparison with the PCL nanoparticles. It causes the copolymer to swell and to degrade faster, thus promoting the drug release from the nanoparticles. It can also be seen from Figure 3 that drug release from the TNP was slightly slower than that of UNP. Such a phenomenon may be attributed to slightly smaller particle size of UNP.

**Figure 3:** **The *in vitro *release profiles of paclitaxel-loaded CNP, UNP, TNP.**

#### Uptake of coumarin-6-loaded nanoparticles by Caco-2 and A549 cells

Caco-2 colonic cell line is a widely accepted model to predict the permeability and absorption of compounds in humans [38]. Paclitaxel (Taxol) has been shown to be effective in metastatic lung cancer as a single agent and in combination with other cytotoxic drugs. The fluorescence uptake by the A549 cells could provide a useful model to assess the *in vitro* therapeutic effect of paclitaxel in the various formulations for lung cancer treatment [39,40]. The cellular uptake of coumarin-6-loaded CNP, UNP, and TNP was thus evaluated in this research using Caco-2 cell line as in vitro model of the GI barrier and A549 cell line as model cancer cells. The cellular uptake efficiency of the coumarin-6-loaded nanoparticles by Caco-2 and A549 cells was assayed upon 2-h incubation, and the results are shown in Figure 4.

**Figure 4:** Cellular uptake of coumarin-6-loaded CNP, UNP, TNP by (A) Caco-2 and (B) A549 cells after 2-h incubation.

It can be obtained from Figure 4A that there is an increasing trend in the Caco-2 cellular uptake: TNP > CNP > UNP. The TNP resulted in 1.45-, 1.61-, and 1.67-fold higher cellular uptakes than those of CNP, and 1.48-, 1.72-, and 1.72-fold higher cellular uptakes than those of UNP at the incubated particle concentration of 100, 250, and 500 μg/ml, respectively. Figure 4A also shows that the cellular uptake was particle concentration-dependent.

Figure 4B shows that the cellular uptake efficiency of the coumarin-6-loaded TNP by A549 cells is higher than that of CNP and UNP, which is also found to be dose-dependent. The TNP resulted in 1.49-, 1.68-, and 1.93-fold higher cellular uptakes than those of CNP, and 1.31-, 1.36-, and 1.65-fold higher cellular uptakes than those of UNP at the incubated particle concentration of 100, 250, and 500 μg/ml, respectively. The positive surface charge of thiolated chitosan provided the incentive to aid drug delivery, since it is expected to ensure better interaction with the negatively charged cell membrane [31,41,42]. This resulted in increased retention time at the cell surface, thus increasing the chances of particle uptake and improving oral drug bioavailability [43].

Figure 5 shows CLSM images of Caco-2 cells after 2 h incubation with the coumarin-6-loaded 5% thiolated chitosan-modified PLA-PCL-TPGS nanoparticles at 250 μg/ml nanoparticle concentration. The images obtained were (A) the enhanced green fluorescent protein (EGFP, green) channel, (B) the DAPI (blue) channel, (C) the overlay of the two channels. It can be observed from Figure 5 that the fluorescence of the coumarin-6-loaded 5% thiolated chitosan-modified PLA-PCL-TPGS nanoparticles (green) is located in the cytoplasm around the nucleus (blue, stained by DAPI), indicating that the coumarin-6-loaded nanoparticles have been internalized into the cells [44].

**Figure 5:** **CLSM images of Caco-2 cells after 2-h incubation with coumarin-6-loaded 5% thiolated chitosan-modified PLA-PCL-TPGS nanoparticles at 37.0°C.** The cells were stained by DAPI (blue), and the coumarin-6-loaded nanoparticles are green. The cellular uptake was visualized by overlaying images obtained by EGFP filter and DAPI filter: left image from EGFP channel (**A**), center image from DAPI channel (**B**), right image from combined EGFP channel and DAPI channel (**C**).

#### Assessment of modified nanoparticle cytotoxicity

Figure 6 shows the viability of A549 cancer cells after 24-, 48-, and 72-h cell culture with paclitaxel formulated in the CNP, UNP, and TNP, respectively, in comparison with that of the Taxol® formulation at the same 0.025, 0.25, 2.5, 10, and 25 μg/ml paclitaxel dose (*n* = 6). It can be concluded from Figure 6 that all three nanoparticle formulations showed advantages in decreasing the cancer cell viability (i.e., increasing the cancer cell mortality) versus the current clinical dosage form Taxol®, and the TNP can have even better effects than UNP. For example, the A549 cell viability after 24-h incubation at the 10 μg/ml drug concentration was 44.41% for Taxol®, and 28.65% (i.e., a 28.39% increase in cytotoxicity) for TNP. Furthermore, compared with Taxol®, the cytotoxicity of A549 cells was increased by 37.65% (*p* < 0.05, *n* = 6) and 18.72% (*p* < 0.05, *n* = 6) for TNP after 48- and 72-h incubation at 10 μg/ml drug concentration. Such advantages of the nanoparticle formulations may be due to the effects of thiolated chitosan and TPGS component of the nanoparticles in enhancing cellular uptake of the nanoparticles. The advantages in cancer cell viability of the TNP > UNP > the Taxol® formulation is dependent on the incubation time. This may be due to the controlled release manner of the nanoparticle formulation. The advantages in cancer cell viability of the TNP > UNP > the Taxol® formulation is also dependent on the drug concentration. The higher the drug concentration, the more significant effects would be obtained.

**Figure 6:** **Viability of A549 cells.** After 24 (**A**), 48 (**B**), and 72 (**C**) hour cell culture with paclitaxel formulated in CNP, UNP, and TNP in comparison with that of Taxol® at the same paclitaxel dose (*n* = 6).

The advantages in cytotoxicity of the TNP > UNP > Taxol® can be quantitatively analyzed by IC_50_, which can be determined by constructing a dose–response curve. Table 2 shows IC_50_ values of A549 cells after 24-, 48-, 72-h incubations with paclitaxel formulated in CNP, UNP, TNP, and Taxol®, respectively, which are obtained from Figure 6. The data showed that the IC_50_ values for A549 cells were reduced from 2.609, 1.645, and 0.910 to 0.201, 0.122, and 0.106 μg/ml for TNP after 24, 48 and 72 h, respectively. As time goes on, the TNP showed better IC_50_ values and better *in vitro* therapeutic effects for A549 cells than commercial Taxol®. This is because the cumulative release of paclitaxel was only 22.63%, 26.52%, and 32.45% for TNP after 24, 48 and 72 h (Figure 3), respectively, and the release started from zero while the commercial Taxol® immediately became 100% available for the A549 cells in culture. Moreover, the degradation of PLA-PCL-TPGS random copolymer may release the TPGS components, which have synergistic antitumor activity in the presence of antitumor drugs [27,28], thus increasing cancer cell mortality. Hasegawa et al. [45] reported a growth-inhibitory effect of chitosan on tumor cells. The growth inhibition was examined by WST-1 colorimetric assay and cell counting. They also observed DNA fragmentation (which is a characteristic of apoptosis) and elevated caspase-3-like activity in thiolated chitosan-treated cancer cells. Chitosan induced apoptosis via caspase-3 activation in lung tumor cells [45]. Therefore, thiolated chitosan may also increase cancer cell mortality and have synergistic antitumor activity in the presence of antitumor agents and TPGS.

**Table 2:** IC50 of A549 cells after 24-, 48-, 72-h incubation with paclitaxel formulated in the Taxol®, CNP, UNP, and TNP

**Incubation time (h)**	**IC_50_ (μg/ml)**			
	**CNP**	**UNP**	**TNP**	**Taxol®**
24	2.035	0.958	0.201	2.609
48	1.748	0.634	0.122	1.645
72	0.692	0.325	0.106	0.910

#### Ex vivo study

In this study, we used the everted intestinal sac method for measuring the transporting of paclitaxel from the intestinal barrier. Figure 7 shows the amount of paclitaxel transported across the intestinal barrier. As seen in the figure, after 120 min, the amount of paclitaxel transported from the intestinal barrier with TNP and CNP was significantly higher than free paclitaxel. Consequently, on the basis of these results, it was hypothesized that the transportation of paclitaxel across the intestine membrane is low, and the mucoadhesive NPs can increase paclitaxel transport by opening tight junctions and bypassing the efflux pump of P-gp.

**Figure 7:** **Profile of the amount of paclitaxel transported in medium (pH 7.4).** Experiments were carried out in triplicate (*n* = 3).

## Conclusions

Three types of nanoparticles were developed from biodegradable self-synthesized PLA-PCL-TPGS random copolymer and commercial PCL for oral delivery of antitumor agents with paclitaxel employed as a model drug, including CNP, UNP, and TNP. The design of the nanoparticle matrix material was made to take full advantages of TPGS in nanoparticle fabrication process such as high emulsification effects and high encapsulation efficiency, as well as improvement of therapeutic effects such as the reduction of P-gp-mediated MDR and superior antitumor efficacy. Thiolated chitosan could greatly increase its mucoadhesiveness and permeation properties, thus increasing the chances of nanoparticle uptake by the gastrointestinal mucosa and improving drug absorption. The data showed that the thiolated chitsoan-modified PLA-PCL-TPGS nanoparticles have significantly higher level of the cell uptake than that of thiolated chitosan-modified PCL nanoparticles and unmodified PLA-PCL-TPGS nanoparticles. *In vitro* cell viability studies showed advantages of the thiolated chitosan-modified PLA-PCL-TPGS nanoparticles over commercial Taxol® in terms of cytotoxicity against A549 cells. It seems that the mucoadhesive nanoparticles can increase paclitaxel transport by opening tight junctions and bypassing the efflux pump of P-gp. In short, oral chemotherapy by thiolated chitosan-modified PLA-PCL-TPGS nanoparticle formulation is an attractive alternative approach to the treatment of lung cancer.

## Competing interest

The authors declare that they have no competing interests.

## Authors’ contributions

LJ carried out the polymer synthesis, nanoparticle preparation, and cell studies. XL carried out the polymer and nanoparticle characterizations. LL carried out the *ex vivo* studies and participated in the design of the study. QZ conceived the study and participated in its design and coordination. All authors read and approved the final manuscript.

## Authors’ information

LJ, XL, LL, QZ are Ph.D., assistant professor, associate professor, and professor, respectively. All authors are from Tianjin Key Laboratory of Biomaterial Research, Institute of Biomedical Engineering, Peking Union Medical College & Chinese Academy of Medical Sciences.

## References

[B1] ChoyHParkCYaoMCurrent status and future prospects for satraplatin, an oral platinum analogueClin Cancer Res20081461633163810.1158/1078-0432.CCR-07-217618347164

[B2] FengSSMeiLAnithaPGanCWZhouWPoly(lactide)-vitamin E derivative/montmorillonite nanoparticle formulations for the oral delivery of paclitaxelBiomaterials200930193297330610.1016/j.biomaterials.2009.02.04519299012

[B3] KuppensIEBoschTMvan MaanenMJRosingHFitzpatrickABeijnenJHSchellensJHOral bioavailability of paclitaxel in combination with OC144-093 (ONT-093)Cancer Chemother Pharmacol2005551727810.1007/s00280-004-0864-415316750

[B4] SparreboomAVan AsperenJMayerUSchinkelAHSmitJWMeijerDKFBorstPNooijenWJBeijnenJHvan TellingenOLimited oral bioavailability and active epithelial excretion of paclitaxel (Taxol) caused by P-glycoprotein in the intestineProc Natl Acad Sci USA1997942031203510.1073/pnas.94.5.20319050899PMC20037

[B5] WilsPPhung-BaVWarneryALechardeurDRaeissiSHidalgoIJSchermanDPolarized transport of paclitaxel and vinblastine mediated by P-glycoprotein in human intestinal epithelial cell monolayersBiochem Pharmacol1994481528153010.1016/0006-2952(94)90580-07945455

[B6] MarreFSanderinkGJde SousaGGaillardCMartinetMRahmaniRHepatic biotransformation of paclitaxel (Taxol) in vitro: involvement of the CYP3A subfamily in humansCancer Res199656129613028640817

[B7] ShouMMartinetMKorzekwaKRKrauszKWGonzalezFJGelboinHVRole of human cytochrome P450 3A4 and 3A5 in the metabolism of Taxol and its derivatives: enzyme specificity, interindividual distribution and metabolic contribution in human liverPharmacogenetics1998839140110.1097/00008571-199810000-000049825831

[B8] ChenHBZhengYTianGTianYZengXWLiuGLiuKXLiLLiZMeiLHuangLQOral delivery of DMAB-modified paclitaxel-loaded PLGA-TPGS nanoparticles for cancer chemotherapyNanoscale Research Letters20116410.1007/s11671-010-9741-8PMC310233627502629

[B9] IkezoeTHisatakeYTakeuchiTOhtsukiYYangYSaidJWTaguchiHKoefflerHPHIV-1 protease inhibitor, ritonavir: a potent inhibitor of CYP3A4, enhanced the anticancer effects of paclitaxel in androgen-independent prostate cancer cells in vitro and in vivoCancer Res2004647426743110.1158/0008-5472.CAN-03-267715492266

[B10] MalingréMMRichelDJBeijnenJHRosingHKoopmanFJTen Bokkel HuininkWWSchotMESchellensJHCoadministration of cyclosporine strongly enhances the oral bioavailability of paclitaxelJ Clin Oncol2001194116011661118168210.1200/JCO.2001.19.4.1160

[B11] ChenHLangerROral particulate delivery: status and future trendsAdv Drug Deliv Rev19983433935010.1016/S0169-409X(98)00047-710837685

[B12] FlorenceATHussainNTranscytosis of nanoparticle and dendrimer delivery systems: evolving vistasAdv Drug Deliv Rev200150suppl 1S69S891157669610.1016/s0169-409x(01)00184-3

[B13] PandeyRZahoorASharmaSKhullerGKNano-encapsulation of azole antifungals: potential applications to improve oral drug deliveryInt J Pharm200530126827610.1016/j.ijpharm.2005.05.02716023808

[B14] des RieuxAFievezVGarinotMSchneiderYJPréatVNanoparticles as potential oral delivery systems of proteins and vaccines: a mechanistic approachJ Control Release2006116112710.1016/j.jconrel.2006.08.01317050027

[B15] LeeDWPowersKBaneyRPhysicochemical properties and blood compatibility of acylated chitosan nanoparticlesCarbohydr Polym20045837137710.1016/j.carbpol.2004.06.033

[B16] Bernkop-SchnurchAHornofMZoidlTThiolated polymers-thiomers: synthesis and in vitro evaluation of chitosan-2-iminothiolane conjugatesInt J Pharm200326022923710.1016/S0378-5173(03)00271-012842342

[B17] Fernandez-UrrusunoRRomaniDCalvoPVila-JatoJLAlonsoMJDevelopment of a freeze-dried formulation of insulin-loaded chitosan nanoparticles intended for nasal administrationSTP Pharma Sciences19999429436

[B18] KastCEValentaCLeopoldMBernkop-SchnurchADesign and in vitro evaluation of a novel bioadhesive vaginal drug delivery system for clotrimazoleJ Control Release20028134735410.1016/S0168-3659(02)00077-912044573

[B19] SaremiSAtyabiFAkhlaghiSPOstadSNDinarvandRThiolated thiolated chitosan nanoparticles for enhancing oral absorption of docetaxel: preparation, in vitro and ex vivo evaluationInt J Nanomedicine201161191282128998910.2147/IJN.S15500PMC3026577

[B20] PanYLiYZhaoHZhengJMXuHWeiGHaoJSCuiFDBioadhesive polysaccharide in protein delivery system: thiolated chitosan nanoparticles improve the intestinal absorption of insulin in vivoInt J Pharm20022491–21391471243344210.1016/s0378-5173(02)00486-6

[B21] AtyabiFTalaieFDinarvandRThiolated chitosan nanoparticles as an oral delivery system for amikacin: in vitro and ex vivo evaluationsJ Nanosci Nanotechnol200998459360310.1166/jnn.2009.109019928123

[B22] AgnihotriSAMallikarjunaNNAminabhaviTMRecent advances on thiolated chitosan-based micro-and nanoparticles in drug deliveryJ Control Release2004100152810.1016/j.jconrel.2004.08.01015491807

[B23] DintamanJMSilvermanJAInhibition of P-glycoprotein by D-alpha-tocopheryl polyethylene glycol 1000 succinate (TPGS)Pharm Res1999161550155610.1023/A:101500050362910554096

[B24] MaYZhengYLiuKTianGTianYXuLYanFHuangLMeiLNanoparticles of poly(lactide-co-glycolide)-d-α-tocopheryl polyethylene glycol 1000 succinate random copolymer for cancer treatmentNanoscale Res Lett2010571161116910.1007/s11671-010-9620-320596457PMC2893931

[B25] YuLBridgersAPolliJVickerALongSRoyAWinnikeRCoffinMVitamin E-TPGS increases absorption flux of an HIV protease inhibitor by enhancing its solubility and permeabilityPharm Res1999161812181710.1023/A:101893900678010644067

[B26] YoukHJLeeEChoiMKLeeYJChungJHKimSHLeeCHLimSJEnhanced anticancer efficacy of alpha-tocopheryl succinate by conjugation with polyethylene glycolJ Control Release2005107435210.1016/j.jconrel.2005.05.01416081183

[B27] ConstantinouCPapasAConstantinouAIVitamin E and cancer: an insight into the anticancer activities of vitamin E isomers and analogsInt J Cancer2008123473975210.1002/ijc.2368918512238

[B28] NeuzilJTomasettiMZhaoYDongLFBirringerMWangXFLowPWuKSalvatoreBARalphSJVitamin E analogs, a novel group of "mitocans," as anticancer agents: the importance of being redox-silentMol Pharmacol20077151185119910.1124/mol.106.03012217220355

[B29] GuHSongCLongDMeiLSunHControlled release of recombinant human nerve growth factor (rhNGF) from poly[(lactic acid)-co-(glycolic acid)] microspheres for the treatment of neurodegenerative disordersPolym Int2007561272128010.1002/pi.2272

[B30] MeiLZhangYZhengYTianGSongCYangDChenHSunHTianYLiuKLiZHuangLA novel paclitaxel-loaded poly (ε-caprolactone)/pluronic F68 nanoparticle overcoming multidrug resistance for breast cancer treatmentNanoscale Res Lett200941530153910.1007/s11671-009-9431-620652101PMC2894322

[B31] MeiLSunHJinXZhuDSunRZhangMSongCModified paclitaxel-loaded nanoparticles for inhibition of hyperplasia in a rabbit arterial balloon injury modelPharm Res200724595596210.1007/s11095-006-9214-z17372684

[B32] MaYHuangLQSongCXZengXWLiuGMeiLNanoparticle formulation of poly(ε-caprolactone-co-lactide)-d-α-tocopheryl polyethylene glycol 1000 succinate random copolymer for cervical cancer treatmentPolymer2010515952595910.1016/j.polymer.2010.10.029

[B33] BarrWHRiegelmanSIntestinal drug absorption and metabolism. I. Comparison of methods and models to study physiological factors of in vitro and in vivo intestinal absorptionJ Pharm Sci197059215416310.1002/jps.26005902045411337

[B34] HosseinzadehHAtyabiFDinarvandROstadSNChitosan–pluronic nanoparticles as oral delivery of anticancer gemcitabine: preparation and in vitro studyInt J Nanomedicine201271851186310.2217/nnm.12.7022605934PMC3352690

[B35] FlorenceATNanoparticle uptake by the oral route: fulfilling its potential?Drug Discov Today20052758110.1016/j.ddtec.2005.05.01924981758

[B36] NorrisDAPuriNSinkoPJThe effect of physical barriers and properties on the oral absorption of particulatesAdv Drug Deliv Rev1998342–31351541083767510.1016/s0169-409x(98)00037-4

[B37] HariharanSBhardwajVBalaISitterbergJBakowskyURavi KumarMNDesign of estradiol loaded PLGA nanoparticulate formulations: a potential oral delivery system for hormone therapyPharm Res20062318419610.1007/s11095-005-8418-y16267632

[B38] ArturssonPPalmKLuthmanKCaco-2 monolayers in experimental and theoretical predictions of drug transportAdv Drug Deliv Rev200146274310.1016/S0169-409X(00)00128-911259831

[B39] NabholtzJMTonkinKSmylieMAuHJLindsayMAMackeyJChemotherapy of lung cancer: are the taxanes going to change the natural history of lung cancer?Expert Opin Pharmacother20001218720610.1517/14656566.1.2.18711249542

[B40] YanFZhangCZhengYMeiLTangLSongCSunHHuangLThe effect of poloxamer 188 on nanoparticle morphology, size, cancer cell uptake, and cytotoxicityNanomedicine20106117017810.1016/j.nano.2009.05.00419447200

[B41] LeroueilPRHongSMeckeABakerJRJrOrrBGBanaszak HollMMNanoparticle interaction with biological membranes: does nanotechnology present a Janus face?Acc Chem Res20074033534210.1021/ar600012y17474708PMC2551762

[B42] SongCLabhasetwarVCuiXUnderwoodTLevyRJArterial uptake of biodegradable nanoparticles for intravascular local drug delivery: results with an acute dog modelJ Control Release199854220121110.1016/S0168-3659(98)00016-99724907

[B43] BhardwajVAnkolaDDGuptaSCSchneiderMLehrCMKumarMNPLGA nanoparticles stabilized with cationic surfactant: safety studies and application in oral delivery of paclitaxel to treat chemical-induced breast cancer in ratPharm Res200926112495250310.1007/s11095-009-9965-419756974

[B44] ZhangYTangLSunLBaoJSongCHuangLLiuKTianYTianGLiZSunHMeiLA novel paclitaxel-loaded poly (ε-caprolactone)/poloxamer 188 blend nanoparticle overcoming multidrug resistance for cancer treatmentActa Biomater2010662045205210.1016/j.actbio.2009.11.03519969111

[B45] HasegawaMYagiKIwakawaSHiraiMThiolated chitosan induces apoptosis via caspase-3 activation in lung tumor cellsJpn J Cancer Res200192445946610.1111/j.1349-7006.2001.tb01116.x11346469PMC5926722

